RETRACTED

# Early Diagnosis and Prediction of Death Risk in Patients with Sepsis by Combined Detection of Serum PCT, BNP, Lactic Acid, and Apache II Score

**DOI:** 10.1155/2022/8522842

**Published:** 2022-07-19

**Authors:** Shuzhen Suo, Liya Luo, Yongkang Song, He Huang, Xixian Chen, Changbo Liu

**Affiliations:** Department of Critical Medicine, The Fourth Affiliated Hospital of Guangzhou Medical University, Guangzhou 511300, China

## Abstract

In order to investigate the expression levels of procalcitonin (PCT), B-type brain natriuretic peptide (BNP), and lactic acid (Lac) in serum of patients with sepsis, a retrospective analysis is conducted. 80 sepsis patients admitted to the ICU of our hospital from January 2019 to June 2020 are selected, and the application value of these factors combined with Apache II score in early diagnosis and prediction of death risk is analyzed. All patients are classified into survival group (*n* = 57) and death group (*n* = 23), and examined by blood routine. Lac, PCT, and BNP, and the serum PCT, BNP, and Lac levels were compared between the nonsepsis group and the control group. Furthermore, Acute Physiology and Chronic Health Status scoring System II (Apache II) is applied to evaluate the score difference between the sepsis group and the control group. The ROC curve demonstrates that PCT, BNP, and Lac combined with Apache II score can obtain high value for early diagnosis of sepsis. Compared with nonsepsis patients, the scores of serum Lac, PCT, and BNP and Apache II are significantly higher in sepsis patients. It is clearly evident that the combined detection of those indicators is valuable for early diagnosis and prediction of death, and will be suitable for widespread clinical application.

## 1. Introduction

Sepsis is caused by infection and systemic inflammatory response syndrome. Severe trauma, major surgery, shock, burns, and other complications are one of the critically ill patients. Sepsis has become one of the main causes of death in the intensive care unit because it can lead to severe sepsis, septic shock, and multiple organ dysfunction syndrome [1]. According to statistics, there are about 18 million sepsis patients in the world, and more than 200,000 people die of sepsis every year. Therefore, it is of great significance to improve the diagnosis and treatment of sepsis. However, sepsis has obvious heterogeneity and a wide range of pathogens. Its early diagnosis and treatment has become a challenge for ICU [2]. The central link of sepsis is inflammation, which runs through the whole pathophysiological process of patients. The release of inflammatory mediators and the infiltration of inflammatory cells lead to the dysfunction of local tissues and corresponding organs. With further development, it can lead to tissue ischemia, hypoxia, hypoperfusion, coagulation dysfunction, and even death due to septic shock [3]. At present, in clinical practice, a variety of inflammatory markers can be applied to the diagnosis of sepsis. However, the detection of a single marker has certain limitations. Therefore, the combined detection of multiple biomarkers has gradually become one of the general trends of sepsis diagnosis, which is of great significance for the application of treatment schemes and prognosis evaluation [4, 5]. Therefore, this study explored the significance of serum procalcitonin (PCT), brain natriuretic peptide (BNP), and lactic acid (LAC) in patients with sepsis. In addition, the role of acute physiology and chronic health assessment II (Apache II) in early diagnosis and mortality risk prediction of sepsis patients was analyzed.

RETRACTED

The remainder of this paper is organized as follows. In Section 2, the related work is discussed.  Section 3 is the inclusion criteria and Apache II score. The results and analysis is presented in Section 4.  Section 5 concludes the paper with a summary.

## 2. Related Work

Sepsis is a systemic inflammatory syndrome caused by bacteria. Most clinical studies have confirmed that there are multiple infectious foci. Therefore, mastering the pathogenesis and process mechanism of sepsis is of great significance for early diagnosis, timely diagnosis, and treatment, and improving the prognosis of such patients [6]. It is of great significance to detect the expression of Lac, PCT, and BNP in the serum of patients with sepsis and to analyze the related mechanisms and detection in the pathogenesis of sepsis. Thus, it provides a theoretical basis for the clinical diagnosis and treatment of sepsis.

After further exploring the related mechanisms of higher expression levels in sepsis patients, some research works prove that, as a single-copy genetic gene composed of 11 amino acids, PCT is the source of monocytes and macrophages. When the body is infected by external bacteria, a large number of PCT will be produced and macrophages will be released to enhance the immune defense ability, which is lower than the bacterial invasion. However, PCT will not be produced in large quantities after the occurrence of immune diseases. Therefore, PCT can be used as one of the main biomarkers of bacterial infection, and its expression level is also high in sepsis patients [7, 8]. At the same time, the PCT level in patients in the death group was significantly higher than that in the survival group. It indicates that the degree of bacterial infection in the death group is more serious, and the degree of tissue and organ damage under bacterial invasion is higher, resulting in higher mortality [9]. BNP is widely distributed in brain, spinal cord, and heart and lung, and mainly comes from ventricles and human plasma. The main form of BNP is 32 peptides with specific circular structure. It has a circular central structure with 17 amino acid residues composed of two cysteines connected by disulfide bonds, and the extension of N-terminal and C-terminal of one 9-residue and one 6-residue. It is similar to ANP and CNP, but its terminal length and amino acid composition are different. Myocardial ischemia, necrosis, injury, ventricular wall tension, and excessive pressure stimulate BNP synthesis and secretion. In addition, its regulation is mainly at the level of gene expression. The nucleic acid sequence of BNP contains unstable tattat sequence, and its messenger RNA is converted rapidly. This enables BNP to be synthesized instantaneously and explosively. Therefore, it can be suggested that its expression level in sepsis patients is significantly higher than that in nonsepsis patients [10, 11]. Secondly, its higher concentration level in the death group also indicates that the degree of external infection is more serious, and the stimulation of myocardial cells is more intense, thus causing the continuous increase of serum BNP level [12]. Lac is a product of metabolism in the absence of oxygen in human body, and its expression level is relatively low in normal body environment. The sharp increase of serum Lac level may indicate that microcirculation disorders in body lead to tissue and organ ischemia, thus providing material conditions for Lac synthesis. However, a large increase in Lac may indicate that organs and tissues are in the state of extreme ischemia and hypoxia, as well as organ failure, threatening the life and health of patients [13, 14]. Therefore, the increased expression of lac in patients with sepsis may indicate that the shock symptoms of patients with sepsis can lead to low perfusion and hypoxia, resulting in the increase of anaerobic metabolites. As a result, lac levels increased significantly. Detection of serum lac level in patients with sepsis can not only assess the severity of the disease but also effectively predict the prognosis of patients [15–19].

RETRACTED

The Apache II score is widely used as one of the main criteria for the severity of the disease in critically ill patients and can be used to evaluate a variety of severe diseases. In this study, the diagnostic efficacy of Apache II score in the diagnosis of sepsis and the prediction of sepsis death was analyzed by drawing ROC curve by combining it with serum Lac, PCT, and BNP. The results showed high evaluation value in both diagnosis and prediction of death. The specificity of combined detection in the diagnosis of sepsis was 81.20% and the sensitivity was 89.40%, while the specificity of combined detection in the prediction of death was 82.10% and the sensitivity was 87.70%, indicating that it had good diagnostic and prediction value [20–23]. However, the specificity of Apache II score alone in the diagnosis and prediction of sepsis death is relatively low, only 58.4% and 62.2%. After further analysis, the author believes that Apache II, as a scoring standard for clinical evaluation of a variety of critical diseases, is applicable in a wide range, so it is not specific. However, it can be combined with its specific markers in the diagnosis of different diseases, which may have higher diagnostic efficacy. The results of this study demonstrated that compared with the control group, serum Lac, PCT, and BNP were significantly higher in the sepsis group, and the levels of Lac, PCT, and BNP in the death group were significantly higher than those in the survival group (all *P* < 0.05).

## 3. Inclusion Criteria and Apache II Score

### 3.1. Inclusion Criteria and Exclusion Criteria

80 patients with sepsis admitted to ICU of our hospital from January 2019 to June 2020 were retrospectively analyzed and included in the sepsis group. 80 nonseptic patients admitted to ICU in the same period were selected as the control group. According to whether the patients died within 4 weeks, the patients were divided into survival group (57 cases) and death group (23 cases). There were 38 females and 42 males in the sepsis group, aged from 38 to 64 years, with an average of (46.45 ± 8.43) year. The control group included 41 females and 39 males. The age of patients ranged from 37 to 65 years, and the average age was (45.98 ± 8.04) years, which was comparable (*P* > 0.05). The survival group included 29 females and 28 males, aged from 38 to 64 years, with an average of (46.44 ± 8.48) year. The death group included 9 females and 14 males, aged between 38 and 65 years, with an average age of (46.83 ± 8.39) years (*P* > 0.05). All patients in the study have the right to know the determination of the test method, and the research content conforms to the principles of the Declaration of Helsinki.

Inclusion criteria mainly include the following: (1) patients with sepsis met the diagnostic criteria of the international consensus conference on sepsis; (2) suspected patients can be classified according to their physical signs, where A represents fever and body temperature higher than 38.3°C, B represents hypothermia and body temperature is lower than 36.0°C, C represents that the heart rate is greater than 90 beats/minute and exceeds 2 standard deviations, D stands for respiratory rate greater than 30 times/minute, E represents the change of consciousness, F represents severe edema or fluid balance change, and G stands for hemodynamic instability.

RETRACTED

Exclusion criteria mainly include the following: (1) younger than 18 years old; (2) admission time exceeds 24 hours; (3) patients with previous malignant tumors; (4) HIV-positive persons; (5) pregnant women.

### 3.2. Apache II Score

The scale mainly consisted of three parts, including acute physiological score, age score, and chronic health score, respectively. The weight of eye opening, language, and motor response in acute physiological score was 1–6 points, and the weight of other indicators was 0–4 points. The age score was 0 for ≤44 years old, 2 for 45–54 years old, 3 for 55–64 years old, 5 for 65–74 years old, and 6 for ≥75 years old. In the chronic health score, nonoperative/elective surgery, inoperable/emergency surgery, and none of the above conditions were recorded as 2, 5, and 0, respectively, with the range from 0 to 71. The higher the score, the worse the condition of the patients.

5 ml fasting venous blood was collected from all patients in the early morning during hospitalization, and put into a centrifuge with a centrifuge parameter of 3500 r/min and a centrifuge radius of 15 cm for 10 min. After centrifugation, supernatant was separated and stored in a low-temperature environment for testing. The serum Lac level was detected by using a LH-750 automatic biochemical analyzer (manufacturer: Beckman Coulter). A Cobas 6000 Automatic Biochemical immunoassay analyzer (Manufacturer: Roche) was used to detect serum PCT level; BNP expression was detected by the immunofluorescence method, and the detection steps were strictly followed the instructions on the immunokit.

### 3.3. Technical Roadmap

Figure 1 showed the technical roadmap, which expresses the research idea in the form of graphs and reflects the comprehensiveness and integration.

## 4. Results and Analysis

Expression of Lac, PCT, and BNP in serum of sepsis group and control group is illustrated in Table 1, where *P* < 0.05.  Figure 2 shows the comparison of serum Lac, PCT, and BNP expression between sepsis group and control group.

Apache II score in sepsis group was significantly higher than that in control group (*P* < 0.05), as shown in Table 2.

The diagnostic efficacy is shown in Table 3. The ROC curve showed that PCT, BNP, and Lac combined with Apache II score had high value for early diagnosis of sepsis, and the area under the curve was significantly higher than other single tests, as shown in Figure 3.

RETRACTED

Lac, PCT, BNP, and Apache II scores in the death group were higher than the survival group (*P* < 0.05), as shown in Table 4 and Figure 4.

The diagnostic efficiency of each indicator is shown in Table 5. The ROC curve shows that the area under the curve of combined detection for predicting sepsis death is significantly higher than single indicator detection, which has a high predictive value for death, as shown in Figure 5.

## 5. Conclusions and the Future Work

In this paper, a retrospective analysis is conducted to investigate the expression levels of PCT, BNP, and Lac in serum of patients with sepsis. The application value of these factors combined with Apache II score in early diagnosis and prediction of death risk is analyzed. The experimental results show that the scores of Lac, PCT, BNP, and Apache II in serum of sepsis patients are higher than those of sepsis patients, and their expression level is higher in the death group. Combined with the scores of Lac, PCT, BNP, and Apache II, the detection of sepsis not only has higher diagnostic efficiency in early diagnosis of sepsis but also can effectively predict the occurrence of death. Therefore, during the clinical diagnosis and treatment of patients with sepsis, real-time monitoring of Lac, PCT, and BNP levels can master the progress of the patient's condition. This can facilitate the adoption of effective measures to prevent the further development of the disease and effectively improve the prognosis of patients. In the future work, we will further explore the application of combined detection of multiple biomarkers in sepsis and improve the diagnostic accuracy of sepsis. In addition, the clinical effects of antibiotics should be evaluated by more extensive research and their efficacy should be evaluated to improve the diagnosis and treatment of sepsis.

## Figures and Tables

**Figure 1:** Technical roadmap.

**Figure 2:** Comparison of serum Lac, PCT, and BNP expression between the sepsis group and control group.

**Figure 3:** ROC evaluation of the diagnostic value of PCT, BNP, and Lac combined with Apache II scores for sepsis.

**Figure 4:** Lac, PCT, and BNP expression and Apache II score were compared between the survival group and the death group.

**Figure 5:** ROC evaluated the predictive value of PCT, BNP, and lactic acid combined with Apache II score for sepsis death.

**Table 1:** Expression of Lac, PCT, and BNP in serum of the sepsis group and control group.

	Number	PCT (ng/mL)	BNP (pg/mL)	Lac (mmol/L)
Sepsis group	80	12.45 ± 1.24	153.32 ± 43.32	3.64 ± 0.23
Control group	80	0.21 ± 0.04	67.32 ± 21.21	1.03 ± 0.24
*t*		21.241	14.23	6.623
*P* value		<0.001	<0.001	<0.001

RETRACTED

**Table 2:** Apache II scores in sepsis group and control group.

	Number	Apache II (score)
Sepsis group	80	54.23 ± 5.56
Control group	80	32.32 ± 6.34
*t*		7.343
*P* value		<0.001

**Table 3:** Diagnostic performance.

	95% CI	Sensitivity (%)	Specificity (%)	AUC	Cutoff value
Joint detection	0.764∼0.925	89.40	81.20	0.845	—
Lac	0.579∼0.784	67.60	53.20	0.681	1.58 mmol/L
BNP	0.598∼0.816	78.90	65.40	0.707	96.54 pg/mL
PCT	0.629∼0.834	78.60	72.10	0.732	5.32 ng/mL
Apache II	0.609∼0.726	59.60	58.40	0.618	37.67

**Table 4:** Expression of Lac, PCT, and BNP in serum of the survival group and death group.

	Number	PCT (ng/mL)	BNP (pg/mL)	Lac (mmol/L)	Apache II (score)
Survival group	57	11.12 ± 1.42	143.23 ± 38.64	3.01 ± 0.25	51.21 ± 4.52
Death group	23	15.56 ± 2.42	176.34 ± 45.65	3.98 ± 0.22	65.42 ± 3.24
*t*		6.431	12.223	6.673	7.722
*P* value		<0.001	<0.001	0.004	<0.001

**Table 5:** Diagnostic performance.

	95% CI	Sensitivity (%)	Specificity (%)	AUC	Cutoff value
Joint detection	0.882∼0.981	87.70	82.10	0.931	—
Lac	0.738∼0.882	83.30	79.40	0.810	3.65 mmol/L
BNP	0.760∼0.828	78.60	69.30	0.749	163.42 pg/mL
PCT	0.672∼0.829	78.30	78.20	0.751	14.34 ng/mL
Apache II	0.512∼0.684	61.20	62.20	0.598	62.23

## Data Availability

The simulation experiment data used to support the findings of this study are available from the corresponding author upon request.
